# Essential Oils from the Fruits and Leaves of *Spondias mombin* Linn.: Chemical Composition, Biological Activity, and Molecular Docking Study

**DOI:** 10.1155/2022/7211015

**Published:** 2022-08-28

**Authors:** Gertrude Adomaa Asante Ampadu, Jehoshaphat Oppong Mensah, Godfred Darko, Lawrence Sheringham Borquaye

**Affiliations:** ^1^Department of Chemistry, Kwame Nkrumah University of Science and Technology, Kumasi, Ghana; ^2^Central Laboratory, Kwame Nkrumah University of Science and Technology, Kumasi, Ghana

## Abstract

This work focused on characterizing the chemical constituents and evaluating the antioxidant and antimicrobial activities of the essential oils obtained from the fruit and leaves of *Spondias mombin—*a flowering plant of the Anacardiaceae *family*. Essential oils were extracted through steam distillation and characterized by gas chromatography-mass spectrometry. For the fruit essential oil, 35 compounds were obtained, and 25 compounds were identified in the leaf essential oil. The dominant compounds present in the fruit essential oil were (*E*)-ethyl cinnamate (14.06%) and benzyl benzoate (12.27%). Methyl salicylate (13.05%) and heptacosane (12.69%) were the abundant compounds in the leaf essential oil. The antioxidant activity of the essential oils was evaluated via phosphomolybdenum, hydrogen peroxide scavenging, 2, 2-diphenyl-1-picrylhydrazyl (DPPH) free radical scavenging, and thiobarbituric acid reactive substances (TBARS) assays. The total antioxidant capacity of fruit and leaf essential oils was 48.5 ± 0.7 *μ*g/gAAE and 48.5 ± 0.7 *μ*g/g AAE, respectively. The half maximal scavenging concentrations of the essential oils in the hydrogen peroxide; DPPH and TBARS assays ranged from 252.2 *μ*g/mL to 2288 *μ*g/mL. The antimicrobial activity of the essential oils was tested using broth dilution and disc diffusion assays against eight microorganisms. The essential oils exhibited broad-spectrum antimicrobial activity against the microorganisms with minimum inhibitory concentrations of 9.75–50 mg/mL. Also, the zones of inhibition of the oils ranged from 12 mm to 25 mm. The biofilm inhibitory activities of the oils were dose-dependent with BIC_50_ values of 42.49 ± 0.1 mg/mL and 97.34 ± 0.6 mg/mL for fruit and leaf essential oils, respectively. Molecular docking studies revealed that the antibiofilm action of the fruit and leaf essential oils could be due to inhibition of the quorum sensing protein, LasR. The results suggest a possible application of the oils as antioxidant and antimicrobial agents.

## 1. Introduction

Essential oils are aromatic oily liquids made up of mixtures of volatile compounds and usually represent a small fraction of a plant's composition. These oils are strongly scented and have a lower density in comparison to water [1]. The aroma of each oil results from the combination of the aromas of all components, with minor oil constituents, even playing critical roles [2]. Essential oils can be isolated from all plant organs—fruits, leaves, stem bark, twigs, and roots—and are mainly composed of terpenes, fatty acids, phenols, alcohols, ketones, and aldehydes [3]. Essential oils have a wide range of biological activities such as antimicrobial, antioxidant, antifungal, and anti-inflammatory activities, and these activities have been attributed to the individual components in the essential oils. Due to the importance of essential oils, they have wide applicability in the food, cosmetic, and fragrance industries.

Essential oils are able to mop up free radicals and hence suppress the action of reactive oxygen and nitrogen species in various matrices. Free radicals, including hydroxyl, superoxide, and nitric oxide radicals, react with molecules in biological systems, leading to oxidative stress. Oxidative stress can cause damage to biologically relevant molecules such as DNA, proteins, carbohydrates, and lipids and has also been implicated in diabetes and neurological malfunctions [4]. The actions of free radicals also cause lipid peroxidation, and this can lead to a significant reduction in food quality [5]. In general, antioxidants function as radical scavengers and inhibit lipid peroxidation and other free radical-mediated processes. As such, they can protect the human body as well as processed foods from oxidative damage. Butyl hydroxytoluene (BHT) and butylated hydroxyanisole (BHA) are synthetic antioxidants that are widely used in the food industry to overcome the action of some free radicals, yet they have not been wholly received by consumers due to negative perceptions about synthetic chemicals and toxicity [6]. There is therefore a high demand for new agents from natural sources to replace some of these synthetic antioxidants. The use of plant-derived antioxidants, such as those containing phenolic substances like flavonoids and phenolic acids in foods, as well as therapeutic medicine, is gaining much recognition. Essential oil components such as phytol and menthol have also been reported to possess antioxidant properties, making their use a potential route for curbing free radical-mediated challenges.

Essential oils and their components have also shown significant activity against microorganisms. Microorganisms are the major drivers of the emergence and reemergence of various infectious diseases. Microbial resistance to existing antimicrobial agents and the absence of new compound scaffolds in the antimicrobial drug pipelines has prompted an urgent need for innovative solutions to this menace. Resistance to the effects of antimicrobial agents occurs due to microorganisms developing strict mechanisms such as making their cell membrane impermeable to drugs, changing drug target sites, or producing enzymes that may degrade antibiotics. Biofilm formation and spore-forming capacity are additional strategies that help the microorganisms to survive in harsh conditions [7]. In the formation of biofilm, microorganisms rely on quorum sensing (QS). This event enables bacteria to express virulence factors such as pyocyanin and pyoverdine. In *Pseudomonas aeruginosa*, QS is regulated by various proteins that are part of a complex structure. The transcriptional activator protein, LasR, sits at the top of the QS hierarchy as it is a primary protein responsible for the activation of the other QS systems, as well as a key player in biofilm formation and virulence genes activation. Inhibition of LasR could interfere with QS and hence biofilm formation [8]. Downregulation of QS, and thus, inhibition of biofilm formation, has therefore been suggested as an innovative approach to tackle the antimicrobial resistance menace. Antimicrobial drugs that interfere with QS and impede biofilm formation are therefore desired. Essential oils, such as those obtained from *Chrysophyllum albidum* and *Synsepalum dulcificum*, have been shown to possess antimicrobial and antibiofilm activities [9, 10]. Essential oil constituents such as p-cymene, thymol, eugenol, and carvacrol have also been shown to possess antibiofilm and anti-QS activities [11]. Essential oils could therefore be integral in developing new strategies for antimicrobial resistance.

*Spondias mombin* Linn. (*S. mombin*) is a flowering plant that belongs to the Anacardiaceae family. The fruits of the plant have leathery skin and a thin layer of pulp, and this has been used in making jelly, juice, jams, and ice cream. The fruit pulp of *S. mombin* is rich in potassium, magnesium, phosphorus, and copper, and these confer high nutritional and functional value [12]. *S. mombin* fruits are used in local medicinal practices for managing ailments such as stomachache, toothache, diarrhea, cough, sore throat, nausea, leprosy, and fungal infections [13]. It has been reported that extracts from the leaves of *S. mombin* exhibit antimicrobial, leishmanicidal, antiviral, hypoglycemic, and antioxidant properties [14]. A concoction from *S. mombin* leaves is widely used for the treatment of diarrhea, dysentery, stomachache, and inflammation [15]. The leaves are also used in folk medicine for the treatment of several topical and systemic diseases like inflammation of the mouth and throat [16]. The essential oils from *S. mombin* from different countries have been reported in other studies, with marked differences in chemical composition. In Nigeria, both Olufunke and Oladimeji analyzed essential oils from *S. mombin* leaves, and in both cases, terpenes such as *β*-caryophyllene and *γ*-cadinene were the dominant constituents [17, 18]. In Brazil, different studies have reported alkanes and terpenes as the major constituents in *S. mombin* leaf and fruit essential oils [19–21]. Since essential oil composition is influenced by environmental conditions such as temperature and light, and cultivation conditions like soil type and soil properties [22], essential oils from the fruits and leaves of *S. mombin* from Ghana were analyzed in this study. The antioxidant, antimicrobial, and biofilm inhibitory activities of the essential oils were also evaluated in different assays. Molecular docking was used to investigate the interactions between the constituents of the oils and the LasR protein, as a means of shedding light on molecular events that may be implicated in biofilm inhibition. Even though many Gram-positive and Gram-negative bacteria form biofilms, biofilm formation in *P. aeruginosa* is well-characterized and the organism is widely used in many studies as a model biofilm-forming organism [23, 24]. *P aeruginosa* was therefore used in this work to study biofilm and QS inhibition capabilities of the essential oils.

## 2. Methods

### 2.1. Sample Collection

Fruits and leaves of *S. mombin* were collected in August 2020 from a farm at Ahinsan (6°40′04.8″N 1°35′28.6″W) in the Ashanti Region of Ghana. The samples were authenticated at the Herbarium Section of the Department of Herbal Medicine, Kwame Nkrumah University of Science and Technology (KNUST). Voucher specimen identification codes were generated for the fruit (KNUST/HMI/2021/FR002) and the leaves (KNUST/HMI/2021/L013) of the plant, after which specimens were deposited in the herbarium.

### 2.2. Sample Preparation

The fruits of *S. mombin* were washed under running water to remove any debris. The pulp of the fruits was separated from the seeds, placed in plastic bags, sealed, and stored at 4°C till extraction. The leaves were washed and air dried under ambient temperature for about 5 days before extraction. Fruits and leaves of *S. mombin* were subjected to steam distillation using the Clevenger apparatus for 3 hours. The oils were concentrated under a vacuum and dried with anhydrous Na_2_SO_4_. The oils were then weighed, and their respective percentage yields were calculated using

(1) $$\begin{array}{c} \text{\% Yield of oil }=\frac{\text{Mass of oil}}{\text{Mass of sample used}}\times 100. \end{array}$$

### 2.3. Chemical Characterization of Essential Oils

#### 2.3.1. Gas Chromatography-Mass Spectrometry

The composition of the essential oils was analyzed on a gas chromatography-mass spectrometry system (Perkin Elmer GC Clarus 580 Gas chromatograph with a Perkin Elmer (Clarus SQ 8 S) mass spectrometer). The mass analyzer of the system was quadrupole. GC-MS conditions were the same as that reported in earlier works from our group [25, 26]. The total GC-MS run time was 34.5 min.

#### 2.3.2. Compound Identification

To identify the compounds present in the essential oils, the mass spectra obtained from the GC-MS analyses were compared to the mass spectra of compounds housed in the National Institute of Standard and Technology (NIST) and Wiley mass spectra databases. Assignment of compound names was made based on the similarity indices with compounds in the NIST and Wiley repositories used in the GC-MS system, as well as spectral data from some published literature [27]. The relative percentages of the various constituents were expressed as percentages calculated by normalization of the peak area.

### 2.4. Antioxidant Activities

The antioxidant activities of the fruit and leaf essential oils of *S. mombin* were assessed using the phosphomolybdenum, 2,2-diphenyl-1-picrylhydrazyl (DPPH) radical scavenging, hydrogen peroxide scavenging, and inhibition of lipid peroxidation assays.

#### 2.4.1. Total Antioxidant Capacity (TAC)

The phosphomolybdenum assay was used to evaluate the total antioxidant capacity of the essential oils. The method used was the same as that used by Afu et al. [28]. Absorbances were measured on an Analytik Jena Specord 200 Plus (Germany) against a blank solution. The standard drug used in the assay was ascorbic acid. Equation (2) was used to compute the TAC (in ascorbic acid equivalent).

(2) $$\begin{array}{c} \text{TAC}=\text{C}\times \text{V}\times \text{M}\times 100\text{,} \end{array}$$

where *M* represents essential oil mass (g) in the reaction mixture, *V* is the total volume (mL) of the reaction mixture,and C is the concentration of ascorbic acid used (*μ*g/mL).

#### 2.4.2. DPPH Free Radical Scavenging Activity

The method used by Gyei and coworkers was used in assessing the DPPH free radical scavenging activity of the essential oils [25]. Different concentrations of the oils were prepared in 5% DMSO. The total reaction volume was 200 *μ*L (DPPH solution, 0.1 mM, 150 *μ*L, and essential oil, 50 *μ*L). Incubation of the mixture was done in the dark for a period of 30 minutes, followed by absorbance measurements of 517 nm on an Analytik Jena Specord 200 Plus spectrophotometer (Germany). The reaction blank was made by using methanol to replace essential oils in the reaction. Positive control for the assay was ascorbic acid. The DPPH scavenging capacity of the essential oils was calculated using

(3) $$\begin{array}{c} \text{\% DPPH radical scavenged}=\frac{\left(\text{Acontrol}-\text{Asample}\right)}{\text{Acontrol}}\times 100, \end{array}$$

where Asample is the absorbance of the test sample and Acontrol is the absorbance of the blank. The IC_50_ values (extract concentration required to scavenge 50% of DPPH radicals) were obtained from a graph of % inhibition against concentration.

#### 2.4.3. Hydrogen Peroxide Scavenging Assay

In this assay, 130 *μ*L of a 5 mM solution of hydrogen peroxide was added to 500 *μ*L of a 1 mM solution of (NH_4_)_2_Fe(SO_4_)_2_·6H_2_O. After this, 3 mL of various concentrations of essential oil or gallic acid (which was used as standard) was added to the mixture and incubated for 30 mins in the dark at ambient conditions. To this mixture was added 1,10-phenanthroline (3 mL, 1 mM). This mixture was uniformly mixed by vigorous shaking, incubated for another 10 mins, and the absorbance of the reaction was measured at 510 nm (Specord 200 Plus, Germany). Water was used in place of essential oils for the blank. Equation (4) was used in computing the percent hydrogen peroxide scavenged.

(4) $$\begin{array}{c} \text{\% Hydrogen peroxide scavenged}=\frac{\text{Atest}}{\text{Acontrol}}\times 100, \end{array}$$

where Atest is the absorbance of the test sample and Acontrol is the absorbance of the blank. The IC_50_ values (extract concentration required to scavenge 50% of hydrogen peroxide radical) were obtained from a graph of % inhibition against concentration [29].

#### 2.4.4. Inhibition of Lipid Peroxidation (TBARS Assay)

For the inhibition of lipid peroxidation assay, Nartey and coworkers' method was employed for this work. The oxidable substrate used for this work was egg yolk. Absorbance measurements were taken at 532 nm (Specord 200 Plus, Germany). Positive controls were butylated hydroxytoluene (BHT) and ascorbic acid. The percentage inhibition of lipid peroxidation was calculated from the absorbance obtained using equation (3). The IC_50_ values (extract concentration required to achieve 50% inhibition of lipid peroxidation) were obtained from a graph of % inhibition against concentration [24].

#### 2.4.5. Data Analysis

Triplicates of all the experiments were made, and the mean and standard deviations were computed. All statistical analyses were made using the GraphPad Prism software 6.0 for Windows (GraphPad Software, San Diego, CA, USA). When *p* < 0.05, it was considered as being statistically significant.

### 2.5. Antimicrobial Activity

#### 2.5.1. Microbial Strains

Microbes used included 4 Gram-positive bacteria (*Staphylococcus aureus* ATCC 29213, *Streptococcus pneumoniae* ATCC 49619, *Bacillus subtillis*, and *Enterococcus faecalis*) and 3 Gram-negative bacteria (*Escherichia coli* ATCC 25922, *Pseudomonas aeruginosa* ATCC 27853, *Klebsiella pneumoniae* ATCC 700603). *Candida albicans* which is a fungus was also used. All microorganisms were obtained from the Department of Pharmaceutics, KNUST. The bacterial strains were cultured at 37°C in nutrient broth overnight, whereas sabouraud dextrose agar was used in culturing *C. albicans*. Microbial cultures were streaked on nutrient agar (Oxoid, UK) plates and incubated at 37°C for 18–24 h. A colony suspension was made in sterile saline, adjusted to 0.5 McFarland standard before further diluting it in sterile double-strength nutrient broth to obtain a concentration of about 2 × 10^5^ CFU/mL.

#### 2.5.2. Minimum Inhibitory Concentrations (MIC)

The broth dilution method was employed in determining the minimum inhibitory concentrations (MICs) of the essential oils. Twofold serial dilution (100 *μ*L) of the essential oil or standard antibiotic (ciprofloxacin) was prepared in sterile 96-well microtiter plates. To each well, 100 *μ*L of appropriate microorganisms in double-strength nutrient broth was added. Following a 24-hour incubation of plates at 37°C, 20 *μ*L of 1.25 mg/mL 3-(4, 5-dimethylthiazol-2-yl)-2,5-diphenyltetrazolium bromide solution (MTT) was added to each well. This was then incubated for 30 min at 37°C. The lowest concentration of test essential oil or standard antibiotic that completely inhibited the growth of the organism as detected by the absence of the purple coloration after MTT addition during a 24-hour incubation period at 37°C was defined as the MIC. Triplicate of each test was performed [30].

#### 2.5.3. Zones of Inhibition

The zones of inhibition of the essential oils were measured in the agar disc diffusion assay. A suspension containing ∼2.0 × 10^5^ CFU/mL of the microorganism was spread on agar media in agar plates. Filter discs were prepared by individually soaking each disc in 30 *μ*L of 30 mg/mL essential oil or 10 *μ*g/mL standard drug. The discs were then impregnated onto the agar plates that had previously been inoculated with the test microorganisms. Discs with solvents, instead of essential oils, were used as the negative control. Ciprofloxacin was used as the standard drug. Plates were incubated at 37°C for 24 hours. Zones of inhibition were measured to assess the antimicrobial activity against each test organism [30].

### 2.6. Biofilm Inhibition

Biofilm inhibitory activities of test essential oils were determined in the crystal violet staining assay. Sterile microtiter plates were filled with 100 *μ*L of MIC and sub-MIC concentrations of test essential oils or gentamicin (used as standard). The bacterial suspension (at 0.5 McFarland standard) was then added to each well to make a total volume of 200 *μ*L. A control experiment, in which solvent was used in place of essential oils, was also set up using the same procedure. The plates were incubated for 24 hours at 37°C, and thereafter, the content of the wells was discarded. This was followed by washing 3 times with deionized water to remove loosely attached cells. Crystal violet (0.1%) was used to stain each well, followed by elution with 30% acetic acid into a new microtiter plate. The absorbances were read at 595 nm (Specord 200 Plus, Germany). Biofilm inhibition was estimated using equation (3). The BIC5_0_ values (drug concentration required to inhibit biofilm formation by 50%) were obtained from a graph of % inhibition against concentration [31].

### 2.7. Molecular Docking Studies

The 3D structure of LasR was obtained from the Protein Data Bank with the PDB code 6V7X [32]. The protein was cocrystallized with the native substrate N-3-oxo-dodecanoyl-l-homoserine lactone and a quorum sensing antiactivator protein AQS1. Prior to docking, the protein was prepared using AutoDockTools-1.5.7rc1. Cocrystallized ligands and water molecules were removed, Gasteiger charges were calculated for atoms, and polar hydrogens were added [33]. The output file was saved in the pdbqt format. Most abundant compounds identified in the fruit and leaf essential oils and compounds that have been reported in the literature to possess antimicrobial activities were used in the molecular docking study. The compounds used from the fruit were (E)-ethyl cinnamate, benzyl benzoate, n-hexadecanoic acid, *cis* vaccenic acid, geraniol, methyl eugenol, terpineol, linalool, a-amyrin, and caryophyllenyl alcohol. For the leaves, hexan-1-ol, 2-methoxy-4-vinylphenol, heptacosane, methyl salicylate, humulene, caryophyllene, longifolene, n-hexadecanoic, and aromadendrene oxide were considered. The 3D structures of the compounds were modeled and optimized in Spartan ‘14 using quantum mechanical methods [34]. To validate the docking protocol in precision docking, the autoinducer AHL was redocked in the ligand-binding domain of LasR. Validation was confirmed based on low RMSD (<2 Å) of the redocked ligand from the orientation of the cocrystallized ligand and the reproduction of observed interactions from the pdb structure [35]. For the compounds, an initial blind docking was performed using PyRx, with an AutoDock Vina extension. This was done to identify the regions on the protein that the ligands preferred to bind. The grid box was defined to cover the whole protein in this blind docking. Compounds that bound in the ligand-binding domain of LasR after blind docking were later subjected to precision docking to probe further into the protein-ligand interactions using the following grid dimensions: center—*X* = 20.0068, *Y* = −3.27362, *Z* = −4.70686, and size—*X*, *Y*, *Z* = 20. Results from the docking were recorded as binding free energy (kcal/mol). Protein-ligand interactions were analyzed using Discovery Studio 2017 R2 client (Dassault Systèmes BIOVIA (Discovery Studio Visualizer) (2017 R2 Client), San Diego: Dassault Systèmes (2017)).

## 3. Results

In this study, essential oils were extracted from the fruits and leaves of *Spondias mombin* using steam distillation in a Clevenger apparatus. Pale yellow oils were obtained with yields of 0.07% for the fruit essential oil and 0.06% for the leaf essential oil. The essential oils were characterized using GC-MS. The total ion chromatograms obtained from the GC-MS analyses for the fruit and leaf essential oils are provided in Figures 1 and 2, respectively. Compounds were identified by comparing the mass spectra obtained in the GC-MS run with available NIST and Wiley spectra libraries. For the fruit essential oil, 35 compounds were identified (Table 1). The dominant compounds present in the fruit and leaf essential oils were (E)-ethyl cinnamate (14.06%) and methyl salicylate (13.05%), respectively. Other compounds present in high amounts in the fruit essential oil were benzyl benzoate (12.27%), n-hexadecanoic acid (8.14%), benzoic acid ethyl ester (5.89%), tetracosane (5.30%), and terpineol (4.61%). For the leaf essential oil (Table 2), heptacosane (12.69%), caryophyllene (6.77%), octacosane (8.54%), and n-hexadecanoic acid (4.91%) were present in high amounts. The class of compounds common to the fruit essential oils were esters (49.05%), acids (14.74%) terpenes (7.93%), phenols (2.85%), alcohols (1.45), ketones (0.34), and alkanes and alkenes (9.59). The leaf essential oil contained alkanes and alkenes (42.70%), esters (14.59%) terpenes (10.34%), phenols (2.93%), acids (6.40), alcohols (5.29%), and ketones (5.78%), as shown in Table 3.

Results from the phosphomolybdenum assay estimated the total antioxidant capacity of the fruit and leaf essential oils as 48.5 and 83.5 *μ*g/g AAE, respectively. The half maximal concentration of the fruit essential oil required for scavenging hydrogen peroxide (IC_50_) was 352.2 ± 0.5 *μ*g/mL and that of the leaf essential oil was 947.2 ± 0.6 *μ*g/mL. The fruit essential oil was therefore a better hydrogen peroxide scavenger compared to the leaf oil. Gallic acid, with an IC_50_ of 9.1 ± 1.3 *μ*g/mL, was used as the standard in this assay. In the DPPH assay, the IC_50_ values for the fruit and leaf essential oils of *S. mombin* were 2112 ± 0.8 *μ*g/mL and 2063 ± 0.7 *μ*g/mL, respectively. Ascorbic acid was used as the standard drug in this assay and its IC_50_ was 14.30 ± 4.3 *μ*g/mL. In the TBARS assay, the fruit essential oil showed better activity in the inhibition of lipid peroxidation compared to the leaf essential oil with IC_50_ values of 1294.0 ± 1.0 *μ*g/mL and 2288.0 ± 0.6 *μ*g/mL for fruit and leaf, respectively. The IC_50_ value of butylated hydroxytoluene (BHT) used in this assay as the standard was 9.2 ± 1.7 *μ*g/mL.  Table 4 summarizes the antioxidant activities of the fruit and leaf essential oils of *S. mombin*.

The antimicrobial activities of the fruit and leaf essential oils of *S. mombin* were evaluated against a panel of microorganisms using both broth dilution and agar disc diffusion methods. The fruit essential oil exhibited zones of inhibition against the tested microorganisms at diameters ranging from 12 mm to 25 mm. The Gram-positive bacteria, *S. aureus* and *S. pneumoniae,* were the most susceptible microorganisms against the fruit essential oil with zones of inhibition of 25 mm and 21 mm, respectively. The fungus, *C. albicans*, recorded a lower zone of inhibition of 12 mm. For *P. aeruginosa*, a Gram-negative bacterium, no zone of inhibition at the concentration of essential oil tested was recorded. The zones of inhibition of the leaf essential oil against *S. pneumoniae* and *K. pneumoniae* were 17 mm and 12 mm, respectively. However, the leaf essential oil showed no zones of inhibition against *S. aureus*, *P. aeruginosa,* or *C. albicans* (Table 5). The MICs for the essential oils ranged from 9.75 mg/mL to 50 mg/mL (Table 6). *S. pneumoniae, K. pneumoniae,* and *E. coli* were the most susceptible organisms to the fruit essential oil with an MIC of 9.75 mg/mL in all cases. A concentration of 19.5 mg/mL of the fruit essential oil was required to inhibit the growth of *S. aureus, B. subtilis, E. faecalis,* and *C. albicans*. Other than *S. aureus* and *P. aeruginosa*, the leaf essential oil was able to inhibit the growth of all tested microorganisms at 23 mg/mL. *S. aureus* was the least susceptible microorganism against the leaf essential oil with its MIC above the concentration tested. The biofilm inhibitory activity of the essential oils was assessed using the crystal violet staining assay with *P. aeruginosa* as the test organism. There was over 40% inhibition of biofilm formation at all concentrations of leaf and fruit essential oils tested. The maximum biofilm inhibition was observed at the MIC for both fruit and leaf essential oils at 62% and 59%, respectively (Table 7). The concentration of the fruit essential oil required for 50% inhibition of biofilm formation (BIC_50_) was 42.49 ± 0.1 mg/mL, which was better than that of the leaf essential oil (BIC_50_ of 97.34 ± 0.6 mg/mL).

Selected compounds present in the leaf and fruit essential oils of *S. mombin* were docked against the LasR protein. This was done to investigate the potential of the docked compounds in modulating the activity of LasR in order to explain the observed anti-biofilm activity. LasR has two domains: an N-terminal ligand-binding domain (LBD)and a C-terminal DNA-binding domain (DBD) (Figure 3(a)). LasR is stabilized and dimerized when its autoinducer 3-oxo-C12-homoserine lactone binds to it. The resultant LasR-AI homodimer complex then attaches to the target DNA promoter and leads to the stimulation of gene transcription. From the crystal structure, the autoinducer interacted with LasR via hydrogen bonding to Trp60, Asp73, Tyr39, Ser129, and hydrophobic interactions with Val76, Cys79, Leu125, and Ala127. Redocking of the cocrystallized acyl-homoserine lactone (AHL) gave a binding affinity of 8.6 kcal/mol. Observed interactions in the redocked structure were hydrogen bond contacts with Trp60, Asp73, Thr75, and Ser129 and hydrophobic contacts with Val76, Cys79, and Leu125. Together, these made up 86% of the reproduced interactions. The root mean squared deviation (RMSD) of the redocked conformation compared to that obtained from pdb was 1.158 Ả (<2 Ả), confirming the docking protocol to be valid for further studies (Figure 3(b)).

The selected ligands were docked to LasR in a blind docking experiment. From the blind docking results, it was observed that 6 compounds from the fruit essential oil were bound at the ligand-binding domain of the protein, while the other 4 compounds bind at regions away from the ligand-binding domain. Compounds that had a binding preference for the ligand-binding domain were benzyl benzoate, (E)-ethyl cinnamate, geraniol, methyl eugenol, terpineol, and linalool (Figure 4(a)). These compounds were subjected to precision docking to probe further into the protein-ligand interactions. Benzyl benzoate formed hydrogen bond contacts with Asp73, Thr75, and Thr115 and hydrophobic interactions with Leu36, Tyr64, Asp73, Val76, Ala105, Leu110, Ser129, and Ile52 with a binding affinity of −10.1 kcal/mol. (E)-ethyl cinnamate also had a binding affinity of −7.8 kcal/mol while establishing hydrophobic interactions with Trp88, Phe101, Ala101, and Leu110. Geraniol established hydrogen bonds with Thr75 and hydrophobic interactions with Leu36, Tyr56, Tyr64, Trp88, Phe101, Ala105, Trp88, and Leu110 with a binding affinity of −6.7 kcal/mol. Methyl eugenol had a binding affinity of −6.8 kcal/mol and formed hydrophobic interactions with Tyr56, Tyr64, Asp73, Trp88, Ala105, and Leu110. With a binding affinity of −7.4 kcal/mol, terpineol established hydrogen bond interaction with Asp73 and hydrophobic interactions with Tyr64, Trp88, Leu110, Ala105, and Phe101. Linalool also had hydrogen bond contact with Ser129 and hydrophobic contacts with Trp88, Phe101, Ala105, and Leu110 with a binding affinity of −6.6 kcal/mol. A summary of the interactions between the compounds and LasR has been provided in Table 8 and Figure 4.

Of the 9 compounds from the leaf essential oil investigated, only 3 compounds (2-hexan-1-ol, 2-methoxy-4-vinylphenol, methyl salicylate) were bound in the ligand-binding domain. The other compounds were bound at different regions of the protein during the blind docking (Figure 5). The three compounds, 2-hexan-1-ol, 2-methoxy-4-vinylphenol, and methyl salicylate, exhibited interactions with residues at the ligand-binding domain with binding affinities of −5.1 kcal/mol, −6.7 kcal/mol and −6.9 kcal/mol, respectively, after precision docking. 2-hexan-1-ol formed hydrophobic interactions with Trp88 and Phe101 while 2-methoxy-4-vinylphenol established hydrophobic interactions with Tyr56, Asp73, Trp88, Phe101, Ala105, and Leu110. Methyl salicylate established hydrogen bond interactions with Tyr56, Thr75, Thr115, Ser129 and hydrophobic contacts with Leu36, Tyr64, Asp73, and Trp88 with a binding affinity of −6.9 kcal/mol, as shown in Table 8 and Figure 5.

## 4. Discussions

Essential oils have been isolated from different plant organs like fruits, leaves, stem bark, twigs, and roots. In this study, steam distillation was utilized in the extraction of essential oils from fruits and leaves of *S. mombin*. The yields of essential oils from the fruits and leaves were 0.07% and 0.06%, respectively. The yields obtained were higher in comparison with the yields reported by de Assis (0.03% and 0.002% for leaves and fruits, respectively) where hydrodistillation was used in the extraction. The yield obtained for the leaf essential oil was also higher than that obtained by Olufunke et al. (0.002%) who subjected fresh leaves to hydrodistillation [17]. The variation in yield may be due to the different methods of extractions used. It has been reported that steam distillation gives a higher yield of essential oils in comparison to hydrodistillation [36]. It could also be due to differences in harvesting seasons and variations in the genetic make-up of the different cultivars [37].

Essential oils are essential in the sense that they contain the essence of the different fragrances and the properties of the plants from which they are obtained [38]. Essential oils are mainly composed of terpenes, fatty acids, phenols, alcohols, ketones, and aldehydes. Gas chromatography coupled with a mass spectrometer (GC-MS) was used to identify the compounds present in the essential oils. The most abundant compound in the leaf essential oil was methyl salicylate. This compound was reported to be present in studies carried out by both Santos and Olufunke [17, 21]. Olufunke and Oladimeji identified caryophyllene as the major component in the leaf essential oil (Table 9) [17, 18]. Even though present in the leaf essential oil in this study, caryophyllene (6.77%) was not the most abundant compound. Other compounds like humulene, naphthalene, and aromadendrene present in this study were also found in the leaf essential oil of *S. mombin* from the other works [20, 21]. For the fruit essential oil, the most dominant compounds were (E)-ethyl cinnamate and benzyl benzoate. Terpineol, which was identified as one of the major components in Santos' work, was present in this study as well. The class of compounds dominant in the fruit essential oil was esters while alkanes dominated in the leaf essential oil. The difference in chemical composition in the fruits and leaves may be due to the nutritional status of the plant as well as genetic and environmental factors [39].

Essential oils exhibit biological properties including antimicrobial, anti-inflammatory, antioxidant, and antimalarial. In nature, essential oils play an important role in the attraction of insects to promote the dispersal of pollens and deter herbivores from feeding on plants by reducing their appetite for plants [40]. The antioxidant activity of essential oils is a biological property of great interest because they may preserve foods from the toxic effects of oxidants [41]. Also, if essential oils can scavenge free radicals, they may play an important role in the prevention of some diseases. The antioxidant activities of the oils were therefore analyzed using various assays (Table 4). The leaf essential oil showed a better total antioxidant capacity compared to the fruit essential oil. In the hydrogen peroxide scavenging assay, the fruit essential oil had a higher scavenging ability than the leaf essential oil. However, the leaf essential oil was observed to be a better DPPH radical scavenger compared to the fruit essential oil. Lipid peroxidation is a complex reaction that can be generated through different pathways [3]. In assessing lipid peroxidation, several lipids' substrates like oils, fats, and fatty acid methyl esters have been used. In this work, the ability of essential oils to inhibit 50% of lipid peroxidation was assessed using the TBARS assay with egg yolk as the substrate. From the results, the fruit essential oil showed a better inhibitory activity compared to the leaf essential oil. Esters and acids have been reported to possess antioxidant activity. Hence, the high antioxidant activity of the fruit essential oil compared to the leaf essential oil may be due to the high composition (63%) of esters and acids in the fruit essential oil. Compounds such as linalool, geraniol, and palmitic acid have been reported to possess antioxidant activity and may be great contributors to the antioxidant activity of the fruit essential oil [42].

The multicomponent chemical composition and complex mechanism of action of essential oils on different bacterial sites make it difficult for bacteria to develop resistance to them [43]. Terpenes such as p-cymene have been shown to cause membrane permeability of bacteria by taking part in membrane swelling. Once the membrane becomes permeable, other essential oil components which target internal organelles (like carvacrol) can then act. This synergy permits the inhibition of the growth of microorganisms [44]. The fruit and leaf essential oils of *S. mombin* showed different activities against tested microorganisms inthe antimicrobial assays. *S. mombin* fruit essential oil showed the greatest activity against *S. pneumoniae* and *K. pneumoniae* with an MIC of 9.75 mg/mL. In addition, high zones of inhibition were observed for these microorganisms in the agar disc diffusion assay. The leaf essential oil did not show any zone of inhibition or MIC against *S. aureus* within the concentrations tested. In general, it was observed that the fruit essential oil exhibited a better antimicrobial activity compared to the leaf essential oil. This may be due to the presence of linalool [45], geraniol [46], and methyl eugenol [47] in the fruit essential oil which have been reported to possess antimicrobial activities. Bacteria can escape the lethal effects of antimicrobials through the formation of biofilm. Therefore, inhibiting biofilm formation is a potential route for eliminating bacteria. The biofilm inhibitory activities of the fruit and leaf essential oils were therefore investigated. From the results, the essential oils showed moderate activities with BIC_50_ values of 42.49 ± 0.1 mg/mL and 97.34 ± 0.6 mg/mL for fruit and leaf essential oils, respectively. It was observed that the biofilm inhibition of both oils was dose-dependent, and inhibition increased with increased concentration. This trend was also observed in a study conducted by Nartey et al. in 2021 [9–26]. Essential oils from *Chrysophyllum albidum*, *Averrhoa carambola,* and several plants have been shown to inhibit biofilm formation. Previous studies have also reported the antibiofilm activities of compounds such as linalool, geraniol, methyl eugenol, and methyl salicylate. These compounds were also identified in the fruit and leaf essential oil and can contribute greatly to its biofilm inhibitory activity. To understand how the compounds in the fruit and leaf essential oils potentially contributed to biofilm inhibition, molecular docking was employed.

Molecular docking was used to predict the binding of the compounds against LasR, a protein that plays a key role in biofilm formation in *P. aeruginosa*. LasR is made up of two protein domains: an amino-terminal ligand-binding domain and a carboxy-terminal DNA-binding domain. In solution, the LasR ligand-binding domain occurs as a homodimer. A long loop, L3, comprising residues Leu40 through Phe51 in the ligand-binding domain, covers the pocket and sequesters the ligand inside the receptor's core, away from the solvent. Residues, such as Tyr56, Trp60, Ser 129, and Asp73, form hydrogen bond contacts with the head group of the autoinducer. A number of hydrophobic residues, including Leu36, Leu40, Ile52, Val76, and Leu125, engage the hydrophobic tail of the N-3-oxo-dodecanoyl homoserine lactone through van der Waals interactions at the other end of LasR's ligand-binding pocket. In the absence of the autoinducer, the loss of these beneficial interactions would presumably result in loop flexibility and subsequent exposure of the buried hydrophobic residues in this pocket to bulk solvent, causing protein aggregation. Similarly, the lack of the autoinducer's interaction with the hydrophobic residues would jeopardize the integrity of the beneficial hydrophobic contacts, resulting in an unstable complex [48].

Of the 10 compounds selected from the fruits for docking, 6 of them had a binding preference for the ligand-binding domain of LasR. Stronger interactions by the six compounds with pocket residues, coupled with their high binding affinities, could probably be responsible for the antibiofilm property of the fruit essential oil. Notably, benzyl benzoate and (E)-ethyl cinnamate, the most abundant compounds in the fruit essential oil, had the highest binding affinities with values of −10.1 kcal/mol and −7.8 kcal/mol, respectively, making them the major probable contributors to antibiofilm action. The other four compounds (geraniol, methyl eugenol, terpineol, and linalool) could collectively contribute to the antibiofilm activity of the fruit essential oil as seen in their binding affinities. From the leaf essential oil, three compounds (2-hexan-1-ol, 2-methoxy-4-vinylphenol, and methyl salicylate) were well accommodated in the ligand-binding domain of LasR while making strong interactions with pocket residues. Observations of the binding affinities of the compounds and their interactions with some key residues in the active site of LasR suggest that the compounds could elicit their biological activity by inhibiting LasR. The abundance of methyl salicylate in the leaf essential oil and its strong affinity for LasR could play a major role in the antibiofilm action, with 2-hexan-1-ol and 2-methoxy-4-vinylphenol fairly contributing to inhibition. The compounds from the fruit essential oil had higher binding affinities for LasR compared to the compounds from the leaf essential oil. This may be the reason the antibiofilm activities of the fruit essential oil observed *in vitro* were better in comparison to the leaf essential oil.

## 5. Conclusions

Essential oils were obtained from the leaves and fruits of *S. mombin* in very good yields. The leaf essential oil was rich in alkanes and alkenes whereas the fruit oil was rich in esters. All essential oils exhibited moderate antioxidant and antimicrobial activities, and this suggests that they could be possible sources of antioxidants in food processing and preservation, as well as antimicrobial agents in the pharmaceutical and cosmetic industries. *S. mombin* fruit and leaf essential oils probably elicit their antibiofilm activity by targeting LasR. Further *in vitro* and *in vivo* studies on the compounds of the essential oils should be conducted to ascertain possible modes by which these compounds act in synergy to elicit the observed activities.

## Figures and Tables

**Figure 1:** Total ion chromatogram (TIC) obtained from the GC-MS run of the essential oil from the fruits of *Spondias mombin*. Compounds were identified by comparison of MS spectra data with NIST and Wiley libraries as well as published literature. The chemical structures of some of the peaks are shown and were drawn with ChemDraw.

**Figure 2:** Total ion chromatogram (TIC) obtained from the GC-MS run of the essential oil from the leaves of *Spondias mombin*. Compounds were identified by comparison of MS spectra data with NIST and Wiley libraries as well as published literature. The chemical structures of some of the peaks are shown and were drawn with ChemDraw.

**Figure 3:** (a) 3D structure of the LasR protein (6v7x) showing the two binding domains. (b) Superimposition of cocrystallized AHL (purple) and redocked AHL (red), RMSD = 1.158 Å.

**Figure 4:** (a) Blind docking of selected compounds from fruit of *Spondias mombin* against LasR. Benzyl benzoate, (E)-ethyl cinnamate, geraniol, methyleugenol, terpineol, and linalool were bound in the ligand-binding domain while n-hexadecanoic acid, *cis* vaccenic acid, a-amyrin, and caryophyllenyl alcohol were outside the ligand-binding domain. (b) 3D interaction of benzyl benzoate with pocket residues of LasR. (c) 3D interaction of (E)-ethyl cinnamate with pocket residues of LasR.

**Figure 5:** (a) Blind docking of selected compounds from leaves of *Spondias mombin* against LasR. 2-hexan-1-ol, 2-methoxy-4-vinylphenol, and methyl salicylate were bound at the active site while heptacosane, humulene, caryophyllene, longifolene, n-hexadecanoic, and aromadendrene oxide were outside the ligand-binding domain. (b) 3D interaction of 2-methoxy-4-vinylphenol with pocket residues of LasR. (c) 3D interaction of methyl salicylate with pocket residues of LasR.

**Table 1:** Chemical composition of fruit essential oils of *Spondias mombin*.

S/N	Name of compound	% Composition	SI (%)
1	Hexanoic acid, ethyl ester	2.07	100.00
2	Benzoic acid, methyl ester	3.98	99.89
3	1, 6-octadien-3-ol,3,7-dimethyl-	2.07	99.89
4	Hexanoic acid, 3-hydroxy-, ethyl ester	3.41	99.78
5	2,4,6-trimethyl-1,3,6-heptatriene	0.60	90.63
6	Benzoic acid, ethyl ester	5.89	99.68
7	Terpineol	4.61	91.12
8	3-cyclohexene-1-acetaldehyde, a,4 dimethyl-	0.45	99.66
9	Geraniol	0.51	99.89
10	Butanoic acid, 3-hydroxy-, ethyl ester	0.65	91.61
11	Benzenepropanoic acid, ethyl ester	3.70	100.00
12	Benzoic acid, 2-methylpropyl ester	0.41	96.99
13	Methyleugenol	2.48	99.37
14	Benzyl methacrylate	0.44	99.87
15	Bicyclo [7.2.0] undec-4-ene, 4,11,11-trimethyl-8-methylene-, [IR-(IR^*∗*^,4Z,9S^*∗*^)]	0.72	99.78
16	2-Propenoic acid, 3-phenyl-, ethyl ester	14.06	99.36
17	3-carene, 4-acetyl-	0.34	97.53
18	Benzene, 1,2,3-trimethoxy-5-(2-propenyl)-	0.58	100.00
19	Caryophyllenyl alcohol	0.66	100.00
20	3,7-cycloundecadien-1-ol, 1,5,5,8-tetramethyl	0.40	99.63
21	1-naphthalenol, decahydro-1,4a-dimethyl-7-(1-methylethylidene)-	0.37	98.81
22	Tetradecanoic acid	0.56	99.55
23	Benzyl benzoate	12.27	100.00
24	E-2-hexenyl benzoate	0.42	90.34
25	Hexadecenoic acid, Z-11-	0.80	97.91
26	n-hexadecanoic acid	8.14	99.33
27	Hexadecanoic acid, ethyl ester	0.61	87.99
28	9-octadecenoic acid(*Z*)-, methyl ester	0.58	97.59
29	*Cis*-vaccenic acid	5.25	99.88
30	9,12-Octadecadienoyl chloride, (*Z*, *Z*)-	3.37	98.55
31	Tricyclo [5.4.3.0 (1,8)] tetradecane-6-one, 4-ethenyl-3-hydrxoxy-2,4,7,14-tetramethyl	0.70	86.49
32	Tetrapentacontane, 1,5,4-dibromo-	0.48	90.97
33	Eicosane	1.79	94.78
34	Tetracosane	5.30	98.80
35	a-Amyrin	0.76	94.88

S/N: compound number in order of elution; %C-% composition of the compound in essential oil SI; similarity index (library search of purity value of a compound).

**Table 2:** Chemical composition of leaf essential oils of *Spondias mombin*.

S/N	Name of compound	% Composition	SI (%)
1	2-hexan-1-ol	2.00	96.15
2	a-methyl-a-[4-methyl-3-pentenyl] oxiranemethanol	1.63	99.88
3	Ethyl 2-(5-methyl-5-vinyltetrahydrofuran-2-yl) prpan-2-yl carbonate	1.54	97.94
4	Methyl salicylate	13.05	99.89
5	Bicyclo [22.1]hept-2-ene, 1,7,7-trimethyl-	3.55	94.19
6	2-methoxy-4-vinylphenol	2.93	98.04
7	Cyclohexane, 1-ethenyl-1-methyl-2,4-bis(1-methylethenyl)-	2.30	98.66
8	Caryophyllene	6.77	99.24
9	Humulene	1.56	95.97
10	1H-cyclopental [1, 3]cyclopropal [1, 2]benzene, octahydro-7-methyl-3-methylene-4-(1-methylethyl)	3.80	90.56
11	Longifolene	2.01	98.38
12	Naphthalene,1,2,3,5,6,8a-hexahydro-4,7-dimethyl-1-(1-methylethyl)	1.35	98.61
13	Aromadendrene oxide-(2)	1.73	94.33
14	Hexadecen-1-ol, trans-9-	1.67	96.56
15	n-hexadecanoic acid	4.91	96.74
16	trans-13-octadecenoic acid	1.49	95.08
17	Octadecane, 3-ethyl-5-(-2-ethylbutyl)-	1.99	91.21
18	Heptacosane	12.69	87.36
19	Hexa-t-butylselenatrisiletane	6.11	95.56
20	3,9-Epoxypregn-16-en-14-ol-20-one, 11,18-diacetoxy-3-methoxy-	5.78	97.30
21	Hentriacontane	3.88	89.06
22	1,2-dipalmitoylphosphatidylcholine	2.82	99.05
23	1,3-bis{[(2Z)-3,7-dimethylocta-2,6-dien-1-yl]oxy}	3.64	89.87
24	Octacosane	8.54	98.79
25	3,5,9-Trioxa-5-phosphaheptacos-18-en-1-aminium,4-hydroxy-N,N-trimethyl-10-oxo	2.26	97.93

S/N: compound number in order of elution; %C-% composition of the compound in essential oil SI; similarity index (library search of purity value of a compound).

**Table 3:** Classification of compounds in the essential oils.

Class of compound	*Spondias mombin* fruit (%)	*Spondias mombin* leaf (%)
Ester	49.05	14.59
Alcohol	1.45	5.29
Acid	14.74	9.20
Ketones	0.34	5.78
Aldehyde	0.45	—
Phenol	2.85	2.93
Terpenes	7.93	10.34
Alkanes and alkenes	9.59	42.70
Others	13.60	9.17

^*∗*^Others: compounds belonging to other classes.

**Table 4:** Antioxidant activities of leaf and fruit essential oils of *S. mombin*.

Sample	TAC^*∗*^ (*μ*g/g AAE)	H_2_O_2_ scavenging activity IC_50_ (*μ*g/mL)	DPPH radical scavenging activity IC_50_ (*μ*g/mL)	TBARS assay^*∗∗*^ IC_50_ (*μ*g/mL)
*S. mombin* fruit	48.5 ± 0.7	352.2 ± 0.5	2112 ± 0.8	1294 ± 1.0
*S*. *mombin* leaf	83.5 ± 0.7	947.2 ± 0.6	2063 ± 0.7	2288 ± 0.6
Ascorbic acid	Nd	Nd	14.30 ± 4.3	Nd
Gallic acid	Nd	9.076 ± 1.3	Nd	Nd
BHT	Nd	Nd	Nd	9.238 ± 1.7

Data represented as mean ± standard deviation, *n* = 3; ^*∗*^TAC: total antioxidant capacity; ^*∗∗*^TBARS: thiobarbituric acid reactive substance assay; nd: not determined (compound not used in that assay).

**Table 5:** Zones of inhibition of *Spondias mombin* fruit and leaf essential oils from the agar disc diffusion assay.

Microorganism	*Spondias mombin* fruit	*Spondias mombin* leaves	Ciprofloxacin
*S. aureus* (+)	25	0	24
*S. pneumoniae* (+)	21	17	22
*K*. *pneumoniae* (−)	19	12	30
*P*. *aeruginosa* (−)	0	0	21
*C. albicans*	12	0	22

+, Gram-positive bacteria; −, Gram-negative bacteria; *C. albicans* is a fungus.

**Table 6:** Minimum inhibitory concentrations of *Spondias mombin* fruit and leaf essential oils.

Microorganisms	*S. mombin* fruit (mg/mL)	*S. mombin* leaf (mg/mL)	Ciprofloxacin (*μ*g/L)
*S*. *aureus* (+)	19.50	>23.00	1.563
*S*. *pneumoniae* (+)	9.75	23.00	3.125
*B*. *subtilis* (+)	19.50	23.00	3.125
*E*. *faecalis* (+)	19.50	23.00	3.125
*P*. *aeruginosa* (−)	25.00	50.00	1.563
*K*. *pneumoniae* (−)	9.75	23.00	1.563
*E*. *coli* (−)	9.75	23.00	3.125
*C*. *albicans*	19.50	23.00	1.563

+, Gram-positive bacteria; −, Gram-negative bacteria; *C. albicans* is a fungus.

**Table 7:** Inhibition of biofilm formation in *P. aeruginosa* by the leaf and fruit essential oils of *Spondias mombin*.

Concentration	% Biofilm inhibition		
	*S. mombin* fruit	*S. mombin* leaf	Gentamicin^*∗*^
MIC	62.89 ± 0.2	59.27 ± 10.3	75.02 ± 19.5
MIC/2	57.10 ± 6.8	51.63 ± 13.4	72.04 ± 16.6
MIC/4	55.50 ± 6.3	49.81 ± 11.5	59.11 ± 9.5
MIC/8	51.59 ± 3.1	47.62 ± 10.1	57.22 ± 9.8
MIC/16	46.90 ± 2.1	42.78 ± 5.1	56.95 ± 10.5
MIC/32	42.50 ± 0.7	38.05 ± 0.5	50.76 ± 6.8
BIC50 (mg/mL)	42.49 *±* 0.1	97.34 *±* 0.6	2.45 ± 1.7

Data presented as mean ± standard deviation, *n* = 3; concentrations of essential oils or gentamicin used were based on their minimum inhibitory concentration (MIC) against *P. aeruginosa*; ^∗^gentamicin was used for comparison purposes.

**Table 8:** Molecular docking results of selected compounds from fruit and leaves of *Spondias mombin*.

Fruit essential oil				Leaf essential oil			
Compound	Binding free energy (Δ*G*)/kcal mol^−1^	Nature of binding interactions		Compound	Binding free energy (Δ*G*)/kcal mol^−1^	Nature of binding interactions	
		Hydrogen bond interactions	Hydrophobic interactions			Hydrogen bond interactions	Hydrophobic interactions
Benzyl benzoate	−10.1	Asp73, Thr75, Thr115	Leu36, Tyr64, Asp73, Val76, Ala105, Leu110, Ser129, Ile52	2-Hexan-1-ol	−5.1		Trp88, Phe101

(E)-ethyl cinnamate	−7.8		Trp88, Phe101, Ala101, and Leu110	2-Methoxy-4-vinylphenol	−6.7		Tyr56, Asp73, Trp88, Phe101, Ala105 and Leu110

Geraniol	−6.7	Thr75	Leu36, Tyr56, Tyr64, Trp88, Phe101, Ala105, Trp88, and Leu110	Methyl salicylate	−6.9	Tyr56, Thr75, Thr115, Ser129	Leu36, Tyr64, Asp73, Trp88

Methyleugenol	−6.8		Tyr56, Tyr64, Asp73, Trp88, Ala105, Leu110				

Terpineol	−7.4	Asp73	Tyr64, Trp88, Leu110, Ala105, and Phe101				

Linalool	−6.6	Ser129	Trp88, Phe101, Ala105, Leu110	^*∗*^Redocked AHL	−8.6	Trp60, Asp73, Thr75, Ser129	Val76, Cys79, Leu125

^∗^AHL is the cocrystallized ligand of LasR. Redocking was done for method validation purposes.

**Table 9:** Comparison of leaf and fruit pulp essential oil composition from different studies.

Source	Constituents (% composition)	Location
*Leaf essential oils*		
Present findings	methyl salicylate (13.05%), heptacosane (12.69%), caryophyllene (6.77%), octacosane (8.54%), and n-hexadecanoic acid (4.91%)	Ghana
Oladimeji et al. 2016 [18]	Beta-caryophyllene (27.875%), gamma-cadinene (12.292%), alpha-humulene (8.074), beta-cadinene (7.785), caryophyllene oxide (6.945)	Nigeria
Ednaldo et al. 2016 [20]	Octadecane (43.51), heptacosane (21.98), hexa-triacontane (15.37), Tetracosane (8.62), 4-hydroxy-4-methyl-2-pentanone (6.41)	Brazil
Santos 2017 [21]	Phytol (11.10%), caryophyllene (9.21%), *δ*-cadiene (5.99%), *α*-humulene (5.25%), *α*-cadinol (3.51%)	Brazil
Olufunke et al. 2003 [17]	*β*-caryophyllene (19.99%), *δ*-cadinene (9.07%), *α*-humulene (6.67%), ℘-muurolene (5.45%), *α*-gurjunene (4.27%)	Nigeria

*Fruit essential oils*		
Present findings	(E)-Ethyl cinnamate (14.06%), benzyl benzoate (12.27%), n-hexadecanoic acid (8.14%), benzoic acid ethyl ester (5.89%), tetracosane (5.30%)	Ghana
Ceva-Antunes et al. 2003 [19]	Myrcene (41.1%), â-phellandrene (8.5), ethyl hexanoate (4.9), butyl butyrate (3.9), camphene (2.5)	Brazil
Santos 2017 [21]	*β*-caryophyllene (26.17%), *α*-humulene (14.65%), (E, E)-*α*-farnesene (12.13%), *α*-terpineol (11.24%), *α*-copaene (4.53%)	Brazil

## Data Availability

All data generated or analyzed during this study are included within the article.
